# Integrating Fuzzy Multiobjective Programming and System Dynamics to Develop an Approach for Talent Retention Policy Selection: Case on Health-Care Industry

**DOI:** 10.1155/2023/5934523

**Published:** 2023-02-18

**Authors:** Chia-Lun Lo, Ya-Han Hu

**Affiliations:** ^1^Department of Health-Business Administration, Fooyin University, Kaohsiung 831301, Taiwan; ^2^Department of Information Management, National Central University, Taoyuan 320317, Taiwan

## Abstract

The demand for medical services has been increasing yearly in aging countries. Medical institutions must hire a large number of staff members to provide efficient and effective health-care services. Because of high workload and pressure, high turnover rates exist among health-care staff members, especially those in nonurban areas, which are characterized by limited resources and a predominance of elderly people. Turnover in health-care institutions is influenced by complex factors, and high turnover rates result in considerable direct and indirect costs for such institutions (Lo and Tseng 2019). Therefore, health-care institutions must adopt appropriate strategies for talent retention. Because institutions cannot determine the most effective talent retention strategy, many of them simply passively adopt a single human resource (HR) policy and make minor adjustments to the selected policy. In the present study, system dynamics modeling was combined with fuzzy multiobjective programming to develop a method for simulating HR planning systems and evaluating the suitability of different HR policies in an institution. We also considered the external insurance policy to be the parameter for the developed multiobjective decision-making model. The simulation results indicated that reducing the turnover rate of new employees in their trial period is the most effective policy for talent retention. The developed procedure is more efficient, effective, and cheaper than the traditional trial-and-error approaches for HR policy selection.

## 1. Introduction

Population aging engenders changes in population structure. Therefore, in aging societies, increasing attention has been paid to issues such as medical care, medical economics, psychology, and social welfare policies. Because of the low muscle strength and flexibility of elderly people, considerable resources must be spent on their health care [1]. However, the challenges involved in caring for elderly people impose high pressure on health-care staff, which results in a high staff turnover rate. Accordingly, staff turnover is a major problem facing health-care institutions in aging countries.

Traditionally, medical service providers maintain their competitiveness by hiring professional personnel to minimize care risks as well as human errors in instrument or device operation and medication provision [2]; thus, labor constitutes more than 45% of the total cost incurred by medical institutions. Some hospitals use human resource planning (HRP) strategies involving a hiring freeze to achieve cost reduction and profits. Other hospitals even occasionally adopt the lowest standard of labor as a business strategy. However, hospitals cannot predict the number of patient visits. In addition, a sudden increase in the number of staff members leads to an increase in the burden on the original staff; this is because the original staff must mentor the new staff. Some new staff members might also make mistakes because of insufficient experience, which can negatively affect the reputation of the hospital they work for. The medical industry is a labor-intensive industry, and cost reduction attempts involving personnel cuts can lead to reduced medical service quality and endanger patients' lives. In addition, a high number of adverse events can occur in a high-burden environment, which increases the rate of human resource (HR) loss. Therefore, cost reduction strategies in the medical industry are associated with moral dilemmas.

Medical institutions must adopt flexible strategies to achieve effective team building and avoid brain drain. In particular, medical institutions can secure their competitiveness by hiring sufficient personnel. Furthermore, when designing HRP strategies, HR planners must consider internal and external factors to ensure that develop comprehensive HR plans and system policy evaluation models from an organizational system perspective.

In the health-care field, root cause analysis (RCA) is one of the most common methods for systematic policy evaluation. RCA is based on secondary data and analysis data obtained through discussions among individuals with different subjective judgments and professional backgrounds [3]. Therefore, RCA can only produce a consensus decision instead of an objectively correct answer [4]. Moreover, the results of the root cause explanations might differ over time. Thus, it is not suitable for HRP issues. HRP is a complicated process and can be defined as a systematic analysis of HR needs to ensure that adequate numbers of employees with the required skills are available at a given time [5]. Several studies have used statistical techniques and mathematical models to forecast HR demand and supply and to execute HRP. However, because of their fundamental limitations, these techniques and models cannot be used for dynamic structural analysis and the identification of delayed feedback effects. Actions undertaken on the basis of inaccurate demand forecasts can occasionally produce results that are contrary to the intended ones. Thus, a systematic tool that can consider complex and dynamic factors must be developed for evaluating HRP policies [6].

In the system dynamics (SD) approach, features such as feedback delays and nonlinear relationships are considered for accurately determining the HR demand and supply. Accordingly, SD modeling is suitable for studying the behavior of a dynamic HRP system [6]. The system dynamics (SD) approach can deal with forecasting inaccuracies and potential mismatches and towards understanding and policy design, which use dynamic features such as feedback delays and nonlinear relationships are considered by very few modelers to deal with HR demand and supply uncertainties. In order to study the behavior of a dynamic HRP system, SD modeling is an appropriate tool.

Several uncertain factors influence the medical actions or administrative decisions taken in a health-care institution. Furthermore, such an institution can have multiple goals related to medical personnel, patients, insurance, and the institution. An SD model considers internal and external factors that affect a system and decreases the percentage of wrong decisions; such a model can thus be beneficial for such institutions. Nevertheless, administrative decisions are complex. Therefore, a fuzzy model can facilitate the task of identifying appropriate administrative decisions. In the medical field, no closed-form solution is generally available for the problem of determining appropriate administrative decisions. The most reasonable approach for administrative decision-making in the medical field involves creating a fuzzy set of multiple decision parameters to determine the optimal decision for achieving a goal. Accordingly, the present study combined SD modeling and fuzzy multiobjective programming (MOP) to develop an HRP system for evaluating the appropriateness of different HR policies in a health-care institution. The SD approach was adopted to create complex and nonlinear models to determine causal feedback relationships [6].

Several studies have adopted SD approaches that entail the consideration of an entire system for analysis. Nonetheless, according to our search of the PubMed database, no study has adopted SD modeling for analyzing nursing talent retention policies in medical institutions. Hence, the present study applied SD modeling to examine the suitability of different labor policies in medical institutions; the study also adopted a hybrid modeling approach to simulate the number of patients that can be accepted in the event of changes in the number of nursing personnel.

## 2. Literature Review

The medical industry is a labor-intensive service sector; thus, HRP is essential in this industry. In general, approximately 30% of the personnel in an acute hospital are nursing staff members. Nurses thus constitute the main personnel in hospital operations. In modern medical treatment procedures, nurses must provide highly professional care to patients. A lack of sufficient nursing staff for posttreatment care might lead to high risks of patient relapse. Thus, nursing staff members play crucial roles at every level in medical institutions.

In general, a higher ratio of nursing staff to patients is associated with superior patient recovery [7, 8]. However, nursing jobs are highly exhausting, and nursing staff must spend considerable time interacting with and satisfying the demands of patients or their families; these requirements impose a high burden on nursing staff members. Consequently, medical institutions experience a high turnover of nursing staff [9]. According to Waldman et al. [10], Most of the hospital staffs are nursing personnel; therefore, the turnover cost for nursing personnel accounts for approximately thirty percent of the total turnover cost. A study indicated that more than 20% of the nursing staff in hospitals had the intention of quitting their job each year in general [11]. A shortage of nursing staff can considerably increase patient mortality rates [12, 13] and in-hospital infection rates [14]. Moreover, a lack of adequate nursing staff might lead to insufficient preservice training and evaluation skills, which result in communication disruptions and thus medical adverse events, including falls [15], medication or transfusion errors [16], treatment delays, complications during or after surgery [11, 17], and prolonged hospital stays [11].

According to Chiu et al. [18], the cost of training a new registered nurse is US$15,825 in the U.S. In addition, insufficient nursing experience results in productivity reduction, the estimated cost of which is US$5,245–US$16,102; it also engenders medical adverse events, which are also associated with a high implicit cost. Therefore, planning strategies for hiring nursing personnel constitute a crucial component of the overall labor planning process of hospitals. The insufficiency of nursing staff is a problem faced by hospitals worldwide [18].

Hospital managers must develop suitable incentives to increase nursing staff retention. However, if managers adopt only salary hikes as a strategy for nursing staff retention, their hospitals would experience high operational pressure because their expenses would increase while their income would remain limited by health insurance systems. Failure to address the problem of nursing staff turnover might lead to a deterioration in nursing quality, which would lead to patients providing poor reviews regarding the hospital. Poor reviews can result in a sharp decrease in hospital income. In Taiwan's insurance payment system, nursing expenses are included in hospital expenses. The salary covered by this system for each nursing personnel is less than $20,000. Thus, hospitals can reduce their nursing expenses only by reducing the number of nursing staff employed [19], hiring contracted staff instead of employees, adopting a working-hour-based salary system, and not recruiting new staff even when vacancies exist. Decreases in the ratio of nursing staff to patients result in staff demoralization and thus high turnover rates. Therefore, hospitals should employ a suitable number of nursing staff such that they minimize expenses while maintaining high health-care quality.

HR quality is more important than HR quantity in most of the industries [20], including the medical industry. Health-care staff members typically differ in terms of literacy, health-care capability, and service quality. Therefore, “clinical advancement systems” have been developed in the nursing industry. Continual on-the-job training can help nursing staff to improve their nursing skills, knowledge, and self-growth, thus increasing their service quality. The current clinical advancement system in Taiwan is based on Benner's theoretical structure, which comprises five stages of skill acquisition in nursing knowledge: novice, advanced beginner, competent, proficient, and expert. The purposes of this system are to help nursing staff transform from novices to experts through step-by-step learning [21, 22] and to reduce staff turnover by higher job achievement.

Managing turnover is crucial for firms because retaining the best talents is essential to remain competitive in the 21st century. Many HR managers have termed the current era as the era of the war for talent [23]. To address the problem of turnover, numerous studies have attempted to determine the key factors that drive turnover [24–27]. However, health-care staff turnover is a dynamic problem because the interrelationships between the factors that influence it to vary. Furthermore, the assumptions underpinning the models constructed in previous studies for assessing health-care staff turnover might become invalid over time. This can thus engender uncertainties regarding the impact of strategies suggested by such models. Consequently, organizations face high risk in strategy implementation, especially when the implemented strategies are ineffective. Considering these limitations, static decision-making models might be unsuitable for modeling health-care staff turnover because they cannot integrate all the variables of a real situation. The basic assumptions of decision-making models are that criteria and alternatives are fixed a priori and that a decision occurs only once; that is, a decision does not involve spatial or temporal considerations. These assumptions limit the validity of the results of the aforementioned models, especially when parameter values change over time and the decision matrix is not fixed or static. In addition, multicriteria decision-making models for talent retention policy selection focus on the cause-effect relationships between individual factors; hence, these models are not comprehensive. Multicriteria decision-making models also generally cannot provide a complete understanding of the complexity of the problem of talent retention policy selection with respect to human-related factors.

Forrester identified a deficiency in the decision-making process of complex dynamic systems [28]. To overcome this deficiency, he proposed SD modeling tools that allow the refining and simulation of mental models for different decision-making policies. Studies have applied SD to address several management problems and provide decision support for managers in many fields [29–32]. A suitable decision-making model must be able to tolerate vagueness or ambiguity because fuzziness and vagueness are common characteristics of most decision-making problems [33]. Accordingly, fuzzy logic (FL) is an essential way for an effective decision-making model [34–37]. The fuzzy theory is the most commonly used concept for solving problems related to imprecise data and ambiguous human judgments in the selection of a talent retention policy. Fuzzy set theory was created to adapt mathematical tools of logic to different types of uncertainty, such as vagueness and approximation, which are characteristics of natural language and human mental models. FL enables the representation of human knowledge through linguistic IF-THEN expressions, which are typical of approximate reasoning [38]. Moreover, FL can be used to obtain solutions to many real-world problems that involve some degree of imprecision and ambiguity, such as talent retention policy selection. Data shortage, measurement errors, or the subjectivity of human judgment can result in uncertain information exhibiting a fuzzy or stochastic nature. Fuzzy models are commonly used because they address various types of uncertainties.

Hybrid models combine different forecasting methods to estimate policy performance. The main advantage of these models is that they can combine different methods and thus leverage their advantages; nevertheless, verifying the rationality of the approach used to combine such methods is difficult. Moreover, hybrid models are characterized by a long computational time.

The first researchers to integrate FL and SD were Pankaj et al. [39], who proposed a method for the qualitative analysis of causal loops by using fuzzy linguistic uncertainties to incorporate the perceptions and beliefs of the modeler. Their motivation was based on the understanding that natural language is the optimal means of expressing the relationships between variables in human mental models. This perception is also the reason behind the development of most hybrid models. Several studies have integrated FL into SD models so that they could consider fuzzy parameters (i.e., their relations, arithmetic, or soft descriptions) when data are unavailable or are not sufficiently credible or when certain parameters exhibit fuzziness [40–42]; these studies did not use FL to define policies to control the developed SD models but instead used it to handle the uncertainty in some model parameters. These models were controlled through a classic approach entailing the use of crisp parameters. Song et al. [43] and Orji and Wei [44] have used SD models to simulate alternative scenarios and then ranked them through MOP. Similarly, Chang and Ko [45], Xu et al. [46], and Wu and Xu [47] have used MOP to control each step of an SD model. This approach is similar to the methodology proposed in this study in that the controller is completely dissociated from the model to be controlled in both approaches. Sabounchi et al. [48] used FL to model decision rules in an SD model of users' transportation preferences.

On the basis of the preceding literature on the combination of FL with SD, we can determine that no study has combined FL with SD modeling for the selection of talent retention policies. Accordingly, the main aim of this study was to design a multiobjective FL-based SD method to handle constraints and uncertain parameters in the evaluation of talent retention policies.

## 3. Methodology

The SD approach is based on systems thinking and is aimed at facilitating learning tasks in complex, feedback, multiloop, multistate, and nonlinear systems in which humans live [49]. It involves using systematic thinking tools to modify mental models repeatedly for implementing reflective learning. Sterman [50] suggested that the SD approach is the best method for resolving complex and dynamic problems. An SD model that considers the interrelationships between internal and external factors can provide specific information related to a complex and dynamic problem and then provide suggestions for the perfect strategic decisions for solving the problem, which would be helpful for managers. In this study, we used the general modeling method proposed by Forrest [51]. SD models are designed to determine the structure of a complex system through the comprehension of concepts such as feedback, stocks, flows, time delays, and nonlinearity [52]. The major components of an SD model include stocks, flows, rates, and auxiliar. Time delay is the most crucial factor in an SD model.

### 3.1. Case Study and Problem Specifications

We conducted a case study on a private and not-for-profit metropolitan hospital in the North of Taiwan. Although this hospital is not a medical center, it is the largest institution with the most beds in the area it is located. The hospital adopts a performance-oriented administrative culture. Various performance management systems have been implemented in this hospital for various posts. Consequently, this hospital is far ahead of the other hospitals in the area in terms of financial performance in the health insurance application. However, the hospital is located in a remote area; thus, it encounters difficulties in retaining personnel. Problems related to HR outflow exist for all the positions in the hospital. Although each hospital employee signs a contract when accepting their job offer, they usually choose to leave the job when their contract expires. Despite improvements in the transportation infrastructure that have removed geographic constraints between the rural area in which the hospital is located and the nearby urban area, employees who remain with the hospital after their contract period are usually locals. In addition, the hospital is a leader in the medical industry; thus, to compete with hospitals in urban areas in attracting talents, it has raised the salaries of its employees, which has led to an increase in its operational costs. Consequently, the net profits of the hospital have decreased within a very short period. However, the hospital still has been unable to solve the problem of HR outflow. Other hospitals that are located in the same area and are of the same level as the case hospital are mostly public institutions or associated with a religious organization, and they have a strong focus on services (e.g., integrated delivery system). Employees of these other hospitals work there because they share altruistic ideals. Thus, these other hospitals need not increase the salaries of their personnel to remain competitive with hospitals located in urban areas. The national health insurance (NHI) system in Taiwan has been adjusted to the managed care-related related policy in recent 20 years. Hospital income cannot be increased without limitation; however, HR costs are still very high.

In this study, the SD modeling process involved five essential steps [53]: (a) problem articulation (boundary selection), (b) dynamic hypothesis formulation, (c) simulation model creation, (d) testing, and (e) policy design and evaluation. The information used for the study was collected from archival records and interviews with health-care personnel, namely, five health-care managers and two directors in the nursing department of the case hospital. Moreover, five strategies were considered as alternative talent retention policies for assessment.

### 3.2. Causal Loop Diagram

The first step in developing an SD model is to define a causal loop diagram. Causal loop diagrams are useful for identifying the feedback loops involved in a process and for representing the feedback structures of systems. The developed SD model captures the relationships between all nodes, including patients, medical staff, hospitals, hospitals' HR policies, and total hospital expenses, to define the system boundary. In this study, the causal loop diagram for the problem of talent retention policy selection focused on nursing staff duty, work pressure, and external information disclosure criteria.

The causal loop diagram described the five aforementioned talent retention policies with respect to the three criteria (nursing staff duty, work pressure, and information disclosure criteria). The developed SD model assumes that when the hospital recruits a new staff member, the workload in the team increases, resulting in this or other staff members resigning and leaving the system; this represents a sequential process, with the new staff member being the first point (stock) of the sequence. The rate of stock inflow was determined. This study set the system boundary on the basis of relevant internal factors, including the number of patients and care staff members; external factors, including population served by the hospital, number of other competing hospitals, insurance budget, and hospital administration policy. The problem specification and the causality of the overall system are described as follows.

Most medical utilization models consider the mutations of epidemic diseases and special health check-ups, but these items are not covered by insurance systems. Medical staff members experience work-related stress when their hospitals adopt new technologies that are challenging to operate. Thus, medical institutions must frequently retrain their staff members to improve their health-care provision skills, which can reduce their work-related stress. Moreover, new employees increase the burden and stress exerted on existing employees because they are unfamiliar with their job processes; the high proportion of new employees (with 30% of front-line staffs of the hospitals being new employees) can be attributed to the high turnover rate of health-care personnel. Because of the burden and stress induced by new employees, staff morale is relatively low, and the health-care quality decreases; this leads to the resignation of existing personnel, thereby creating a vicious circle. A decrease in health-care personnel leads to a decrease in health-care supply and an increase in the duty ratio (health-care demand/health-care supply), which imposes extra stress on front-line personnel and leads to a further increase in their turnover rate. The expansion limits set for hospitals by the health-care insurance organization when preparing its budget are based on regional totals and the calculation method of point values. Hospitals frequently adopt incentive measures to increase their market share, and these measures often increase their medical resource consumption and expenses. Moreover, the performance system causes increases in the number of patients and the personnel workload. Medical institutions require a prolonged time to recruit new employees in response to increases in workload. Failure to promptly recruit new employees to take up the excess workload leads to stress among existing personnel, and this ultimately increases their turnover rates; the high turnover increases the institution's expenses. In summary, factors such as population aging lead to an increase in the demand for medical services; nevertheless, the supply of such services is limited and is governed by the total number of people paying insurance premiums. Thus, relevant authorities have developed many policies to restrain the growth of hospitals' expenses and reduce their expenses if possible. However, as displayed in the causal loop diagram, a reduction in hospital expenses might increase health-care risks. When insufficient health-care personnel is available to meet patients' health-care demands, some balancing policies must be adopted to ensure that patients' rights and treatments are not negatively affected.

To estimate the performance of different strategies for workload reduction, factors related to revenue sustainability, such as the total insurance budget/cost associated with a particular nursing staff member, should be considered first. The performance of different strategies was estimated by experts by using fuzzy questionnaires and real data collected from the case hospital. The following five HR balancing strategies were evaluated in this study [6].

#### 3.2.1. Policy 1: Changing the Care Model

Policy 1 involves replacing the original primary nursing model with a functional care model. However, although the adoption of the functional care model can temporarily increase efficiency, the root problem of insufficient medical supply still exists. Thus, personnel are still under stress and may eventually resign. Policy 1 might help balance the causal loop over the short term; however, it can also lead to a long-term time delay effect. Therefore, policy 1 has unsuitable effects over the long term.

#### 3.2.2. Policy 2: Increasing Working Hours

Policy 2 involves making health-care personnel work overtime. The number of patients and the workload of long-term care institutions are somewhat fixed, and employees often work overtime in these institutions. However, health care is a persistent job. The tasks involved in each shift must be handed over to the person working the next shift, and many varied tasks are conducted in hospitals. In the short term, increasing working hours can increase the medical supply; however, over the long term, overtime might lead to high turnover rates and thus a time delay effect.

#### 3.2.3. Policy 3: Increasing the Number of Patients Attended to by Each Health-Care Professional

Patients must be cared for even when the supply of manpower is insufficient. Patients cannot be discharged because of an inadequate workforce. Therefore, the number of patients assigned to a single health-care personnel is increased to meet care needs. When the number of health-care employees in a hospital decreases, the duty rates for the remaining employees are increased because the number of patients is unchanged. According to the literature, when the number of patients to be cared for by each health-care professional decreases by 1, the corresponding health-care quality, staff morale, and job satisfaction decrease [12, 14], which results in personnel resignations over the long term. Thus, policy 3 results in a time delay effect over the long term.

#### 3.2.4. Policy 4: Increasing the Number of Care Staff Members

Although an upper bound exists for the number of patients assigned to each health-care personnel (i.e., a maximum of 2.5 beds assigned to a single health-care personnel), hospitals usually consider their entire staff, including those in administrative units, outpatient units, and other special units, when evaluating the number of patients to assign to their personnel. Thus, the actual number of available personnel is different from the reported number of personnel. Consequently, when the number of care personnel decreases, the workload of the remaining personnel increases considerably. Because the HR departments of hospitals consider only the total number of personnel as a basis for recruitment, the number of care personnel hired might be insufficient, which negatively affects the provided health care and increases the workload of health-care personnel. This also engenders a time delay effect.

#### 3.2.5. Policy 5: Reducing the Number of Available Beds

Under policy 5, the numbers of beds and health-care personnel are regulated according to the ratio of beds to total personnel. When the number of personnel is insufficient, some wards can be closed or the bed availability can be reduced. The removal of beds results in a decrease in long-term medical demand. However, this measure does not help reduce the immediate medical demand or the number of person-days of hospitalization. Consequently, the workload might increase in the short term. The main problem associated with removing beds is that hospitals cannot turn away patients, and reducing the number of beds would result in complaints about long waiting periods for hospitalization. Thus, the stress on employees might increase over the long term, which is a time delay effect.

On the basis of the preceding analysis, this study established a diagram to demonstrate the possible reason for the high turnover of health-care staff (especially nursing staff) and to outline policies that can be adopted by health-care institutions to address the problems caused by the high turnover, as presented in Figure 1. The next section presents the stock and flow diagrams as well as their equations, all of which were used to analyze the relationship of the policies and the stabilize of the HR structure in the case hospital. We attempted to identify a suitable strategy for handling care staff turnover.

### 3.3. Stock Flow Diagram

The proposed SD model combines HR demand and HR supply to evaluate HR policies. On the basis of the aforementioned causal loop diagram, we created a stock-flow diagram. Subsequently, the dynamic equations for each element in the stock flow diagram were added to the developed SD model.

The ultimate purpose of an SD model is to help a manager simulate the influences of management decisions on system growth and stability in a management system. The manager can then develop measures or policies to improve system performance. Therefore, only the manager can decide whether the SD model helps improve the actual management performance.

In the proposed methodology, the system to be governed (modeled using SD stock and flow language) is separated from the human decision-making system (policies). A stock node (symbolized by a rectangle) represents a point where content can accumulate and deplete. A flow node (symbolized by a valve) is a rate of change in a stock node, and it represents an activity, which fills in or drains the stock node. An auxiliary node or a constant node can store an equation or a constant. Finally, the connectors, represented by simple arrows, are the information links representing the cause and effects within the model structure; the double arrows represent physical flows. Double lines across the arrows indicate time-delayed information.

We created our stock flow diagram for the health-care subsector by using the number of care staff members and the workload information. Providing health care to patients is a skill. The experience of health-care personnel influences the quality of the care they provide and their risks of making errors during care provision. According to the HRP model proposed by Nkomo, experience differences between personnel should be considered to reduce errors in evaluations. Therefore, the present study referenced the skill acquisition model developed by Hubert and Dreyfus to design an HR classification structure [54]. However, interviews with administrators from the case hospital indicated that the developed five-level structure was excessively complex. Therefore, we categorized nurses in the second year of their job as advanced nurses, those in the third year of their job as senior nurses, and those holding a position in the administration or nursing department as experts. The stock-flow diagram for HRs in nursing is displayed in Figure 2.

The trial period for each employee in the case hospital is 3 months, and those who pass their trial period become official employees. New recruits are junior nurses, who become senior nurses after gaining 1 year of experience. Every year, the case hospital conducts a survey of employees' willingness to remain at the hospital. Those who wish to resign can be classified into the category of “expected to leave office.” According to the manager of the case hospital, personnel changes after the expiry of contracts are usually related to transfers from a first-line post to another post or resignations due to family needs. As revealed by annual survey data, the turnover rates of the case hospital are 65% and 30% for advanced and senior personnel, respectively.

#### 3.3.1. Calculating Number of Care Staff Members and Workload

To determine HR supply and HR demand, the current number of staff members must be calculated. Moreover, weights should be assigned for various factors for calculation. According to the interviews conducted in this study, the case hospital adjusts its number of job vacancies on the basis of its current HRs. The main recruitment stages are usually implemented after two national exams every year; however, the number of people the hospital has recruited and the number of people it reports to have recruited are two factors that should be considered for calculation. In addition to the workload demand, the number of people of different seniority levels leaving the hospital should be considered during the calculation of the quantity of resources required to fill these vacancies. The time required to find suitable candidates usually differs for different seniority levels. An interviewee stated that finding suitable candidates immediately was impossible. Therefore, in the case of departures, the additional workload was spread among the remaining personnel. Consequently, the weight pertaining to workload could be set to 1.

Because the seniority of first-line health-care personnel might influence their service quality, a suitable weight should be adopted for personnel at each seniority level. Therefore, we set a weight of 1 for senior staff and experts. The interviews also indicated that during the trial period, personnel usually spend their time learning. Moreover, they provide care to patients with simple conditions. After the trial period, personnel are fully integrated into the health-care provision system. Senior staff must spend time teaching new staff in the trial period. Accordingly, we set a weight of −1 for senior staff providing assistance during the trial period. Moreover, directors cannot engage in health care when they are interviewing junior staff. Therefore, we set a weight of 0.8 for directors. Finally, we set a weight of 0.9 for registered nurses who plan to leave the job after the expiration of their contracts. Because the weight of the resignation possibility includes negative numbers, we adopted a setting to avoid negative values.

A higher person-days of hospitalization might lead to higher workloads for health-care staff. However, for calculation, an assumption of a three-shift system (day, evening, and overnight shifts) would be more convenient than a 24 hours way; thus, person-days were converted into hours. The maximum number of patients assigned to each care personnel in the three-shift system was set to 8, 10, and 12 for the day, evening, and overnight shifts, respectively. Moreover, the time required for patient care varies with disease severity. Hence, we also considered disease severity in terms of the Carlson comorbidity index and set the risk ratio to 1.2 [55]. We also set the daily nursing hours to 8 h per day. Because working overtime is highly common in hospitals, a corresponding parameter was added to the system dynamic model.

Health-care workloads might increase because of changes in health-care tasks, and increased workload is a major reason for HR outflow. This time delay factor should be considered before applying any response measures. Thus, the nursing workload ratio was set to 1. A nursing workload ratio higher than 1 indicates excessive workload. The time required to recruit new staff to fill vacancies was set to 6 months. Because the provided health care affects people's health considerably, medical service quality must be considered when assigning jobs. In addition, upper bounds should be set for the workload. Accordingly, the upper bound was set to 12, 15, and 18 patients for the day, evening, and overnight shifts, respectively. The literature reveals that a positive relationship exists between work pressure and HR outflow. This study thus developed an HR outflow function (Figure 3) and a stock-flow diagram (Figure 4) for the analysis of staff workload.

In general, if a manager wishes to make a suitable policy decision, they must consider strategic approaches toward multiple policy objectives. Moreover, they should avoid linear thinking to avoid making wrong decisions. However, determining the best multiobjective policy through humans' limited thinking loops is difficult. Therefore, the MOP model can be used to design different objective functions under a set of constraints for decision-making in systems involving two or more goals.

As mentioned, every system has unique objectives and requirements pertaining to workforce planning. To achieve all objectives and find the best solution, all the adopted systems must be balanced in every loop. Patients generally wish to receive the best (most expensive) service; however, the insurance expense system of a hospital must minimize the hospital's claimed expenses. Therefore, a hospital management system is typically designed to increase the hospital's revenue by maximizing its income and minimizing its costs (the labor cost accounts for the highest percentage of all costs in a hospital). Employees prefer their labor payment to be increased to the highest amount possible. If the labor payment is insufficient, employees' willingness to offer high-quality services might be influenced, which can considerably influence patients' perceptions of the hospital. Thus, optimizing the aforementioned multiobjective parameters through SD modeling can facilitate a more comprehensive policy consideration process. We conducted simulations for the multiobjective optimization model developed in this study by adding insurance and workforce constraints to the model. We also considered the effects of turnover on the balance of possible institutional changes or structural workforce changes. These effects were determined by decision nodes, which were represented by the growth rate of each industry, in the simulations. Some of the constraints used in the baseline scenario are described as follows.

*(1) Population Subsystem*. A strong relationship exists between medical demands and population. We defined the demand subsector and population subsector. Population data obtained from the Department of Statistics, Ministry of the Interior, Taiwan, revealed that by the end of 2013, a total of 458,456 people resided in the county in which the case hospital is located. Among them, 88,112 people (20% of the county population) were aged older than 65 years. Overall, elderly people constitute 11.53% of the population of Taiwan in 2013. Therefore, the aforementioned county has a high population of elderly people.  Table 1 presents the population trend over the past 10 years in this county. Population aging engenders increased medical demand and increased workload for health-care staff.

*(2) Revenue Subsystem*. The Taiwan NHI system is different from those of other countries with a family doctor system. In Taiwan, no appointment system exists for outpatient services; however, moral constraints prevent doctors from declining any patient. Most Taiwanese hospitals have a culture of performance incentives based on physician fees. Therefore, the numbers of patients in Taiwanese hospitals are very high, which leads to high workloads and work pressure for health-care staff. Accordingly, we collected data on the monthly numbers of patients in the case hospital to define our simulation parameters. With regard to medical revenue, the data collected by this study from the case hospital included medical income from inpatient and outpatient services covered by the NHI program, medical income from medical services paid by patients, and nonmedical income. The main revenue source of the case hospital was the income obtained from services covered by the NHI program; information regarding all other sources of revenue was confidential. Therefore, our simulations were related to the services covered by the NHI in the case hospital. Partial revenue data for the case hospital are presented in Table 2.

*(3) Care Provider Subsystem*. The purpose of this study was to analyze the influences of the HRP policies of a medical institution on the outflow of its health-care staff. Thus, the HR supply data used in this study comprised the number of nursing personnel in the case hospital and the number of personnel resigning from the case hospital. We collected monthly data regarding the experience levels of the nursing staff (N–N4) and the number of personnel of each level who resigned from the hospital (including those who resigned and those who could not perform first-line tasks because of different reasons) over a 5-year period. In general, the peak period for nursing staff outflow in the case hospital was determined to be from July to September and from February to April.  Table 3 presents a summary of the number of nursing staff members who resigned from the case hospital over the 5-year period, which increased exponentially.

### 3.4. Fuzzy MOP Model

An MOP model is typically used to maximize or minimize different objective functions under a set of constraints and is essential for decision-making in systems involving two or more goals. In a system for selecting a suitable strategy for health-care talent retention, each subsystem has unique goals, and each item must be optimized to achieve a suitable trade-off among the subsystems. In general, in such a system, the health-care institution's revenue and insurance revenue must be maximized, whereas the HR cost must be minimized. To achieve these goals, system parameters that strongly influence the system output must be identified. Accordingly, we developed an MOP model and applied it to a dynamic system to optimize its parameters. The notations used in this section are listed in Table 4.

#### 3.4.1. Objective Function

*(1) Objective Related to a Health-Care Institution's Revenue*. Health-care institutions are nonprofit organizations; however, they must generate sufficient revenue to operate sustainably. Some health-care institutions have also started commercializing their services. They must earn revenue that at least equals the operating cost and the capitalized cost related to the new investments. In addition, under the influences of an unlimited insurance policy and private patient fees, achieving maximum revenue has become a major objective of most health-care institutions. This objective can be considered the first objective in this study and can be expressed as follows:

(1) $$\begin{array}{c} f_{1}=E_{1}+E_{2}+E_{3}+E_{4}\text{,}\\ E_{1}=G_{1}\left(1+x_{1}\right)+G_{2}\left(1+x_{1}\right)+G_{3}\left(1+x_{1}\right)\text{,}\\ E_{2}=G_{1}\left(1+x_{2}\right)+G_{2}\left(1+x_{2}\right)+G_{3}\left(1+x_{2}\right)\text{,}\\ E_{3}=G_{1}\left(1+x_{3}\right)+G_{2}\left(1+x_{3}\right)+G_{3}\left(1+x_{3}\right)\text{,}\\ E_{4}=G_{1}\left(1+x_{4}\right)+G_{2}\left(1+x_{4}\right)+G_{3}\left(1+x_{4}\right)\text{.} \end{array}$$

*(2) Objective Related to the Insurance System*. Unlimited growth in the global insurance budget is impossible, and this budget influences the economy and civil atmosphere of a nation. Rapid aging in a society engenders increased health-care demand, and a gap between health-care demand and supply is a developmental bottleneck for health-care institutions. Therefore, reducing insurance fees is a major objective of the National Health Insurance Administration (NHIA) of Taiwan, which can be considered the second objective in this study. This objective can be expressed as follows:

(2) $$\begin{array}{c} f_{2}=C_{1}+C_{2}+C_{3}+C_{4}-C_{5}\text{,}\\ C_{1}=G_{1}\left(1+x_{1}\right)a_{11}+G_{2}\left(1+x_{2}\right)a_{12}+G_{3}\left(1+x_{3}\right)a_{13}\text{,}\\ C_{2}=G_{1}\left(1+x_{1}\right)a_{21}+G_{2}\left(1+x_{2}\right)a_{22}+G_{3}\left(1+x_{3}\right)a_{23}\text{,}\\ C_{3}=G_{1}\left(1+x_{1}\right)a_{31}+G_{2}\left(1+x_{2}\right)a_{32}+G_{3}\left(1+x_{3}\right)a_{33}\text{,}\\ C_{4}=G_{1}\left(1+x_{1}\right)a_{41}+G_{2}\left(1+x_{2}\right)a_{42}+G_{3}\left(1+x_{3}\right)a_{43}\text{,}\\ C_{5}=x_{4}\alpha_{1}\text{,} \end{array}$$

where *C*_1_, *C*_2_, *C*_3_, and *C*_4_ represent the global budgets of western medicine consumption, western primary medicine consumption, Chinese medicine consumption, and dental medicine consumption, respectively, at the three hospital levels (medical centers, metropolitan hospitals, and district hospital). Moreover, *C*_5_ denotes the insurance amount saved through any budget control policy.

*(3) Objective Related to the HR Cost*. The expansion of a hospital is limited by the total population in its region and the global budget of insurance fee point calculation systems, which can result in a crowding-out effect. Thus, hospital expenses should be decreased to raise hospital profits; the HR cost accounts for the highest proportion of the total expenses of a health-care institution. However, according to the causal loop diagram, expense reductions might increase the risks associated with patient care. Therefore, the HR cost must be minimized such that patient safety is not compromised. This can be considered the third objective in this study and can be expressed as follows:

(3) $$\begin{array}{c} f_{3}=s_{1}c_{1}+s_{2}c_{2}+s_{3}c_{3}-x_{5}\alpha_{2}\text{.} \end{array}$$

The final item in equation (3) is the NHI claim reduction resulting from the health-care institution's internal adjustment policy.

#### 3.4.2. Constraints

Decision-makers select their preferences for the relationships between factors or variables in an HRP system, and these preferences are then considered as constraints for MOP.

*(1) Constraint Related to the Growth of a Health-Care Institution*. Health-care demands and expenses increase with the growth of the elderly population in an area. However, increases in the use of insurance resources and institution costs must be limited while meeting the health-care demand. Therefore, an upper bound for the growth rate of a health-care institution is a constraint in an HRP system. Moreover, the growth rate of NHI fees must be higher than the development rate of health-care institutions in the relevant country. Accordingly, the constraint for the growth of a health-care institution can be expressed as follows:

(4) $$\begin{array}{c} f_{1}=\frac{\left(E_{1}+E_{2}+E_{3}\right)}{E}\leq d_{1}\text{,} \end{array}$$

where *d*_1_ represents the minimum growth rate of insurance fees.

*(2) Investment Constraints*. Most health-care institutions in Taiwan are nonprofit organizations covered by insurance, which indicates that they have limited income. They cannot invest in other businesses and must use their revenue for their own needs. In general, the manager of a health-care institution must strive to achieve a cost allocation of 33% for each of the following aspects of their institution: HRs, medicines, and utilities. Therefore, the proportion of investment into HRP is limited. Let *d*_2_ and *d*_3_ represent the upper limits of the global budget and HRP budget, respectively; hence, the following equations can be derived:

(5) $$\begin{array}{c} x_{4}\leq d_{2}\text{,}\\ x_{5}\leq d_{3}\text{.} \end{array}$$

*(3) Insurance Source Constraints*. Insurance consumption mainly varies with the age of, health-care literacy of, and medical advice obtained by an individual. Moreover, the density of hospitals in an area and the proportion of the population seeking medical advice in this area govern the consumption of insurance resources, especially after the implementation of the capitation and fee-for-service reimbursement system. To control the growth rate of insurance consumption, the NHIA can set fixed thresholds or constraints to regulate the frequency at which people can seek medical advice and the frequency of hospitalization (e.g., global budget or diagnosis-related group system). Accordingly, the following proportional constraints can generally be applied:

(6) $$\begin{array}{c} b_{11}\leq \frac{a_{1}c_{1}}{a_{1}c_{1}+a_{2}c_{2}+a_{3}c_{3}+a_{4}c_{4}}\leq b_{12}\text{,}\\ b_{21}\leq \frac{a_{2}c_{2}}{a_{1}c_{1}+a_{2}c_{2}+a_{3}c_{3}+a_{4}c_{4}}\leq b_{22}\text{,}\\ b_{31}\leq \frac{a_{3}c_{3}}{a_{1}c_{1}+a_{2}c_{2}+a_{3}c_{3}+a_{4}c_{4}}\leq b_{32}\text{,}\\ b_{41}\leq \frac{a_{4}c_{4}}{a_{1}c_{1}+a_{2}c_{2}+a_{3}c_{3}+a_{4}c_{4}}\leq b_{42}\text{.} \end{array}$$

Moreover, the insurance budget for the current year should be less than that for the previous year. Hence, the following inequality should be satisfied:

(7) $$\begin{array}{c} \frac{f_{2}}{f_{1}}\leq IF\left(1-d_{4}\right)\text{,} \end{array}$$

where IF denotes the insurance fee for the previous year and *d*_4_ is the average rate of increase in this fee.

*(4) Constraint Related to the HR Cost*. The HR cost generally accounts for the highest proportion of the total cost incurred by a health-care institution. Therefore, from an administrator's viewpoint, an increase in HR costs should be minimized. The constraint for the increase in HR cost is similar to that for the increase in insurance resource consumption, and the following inequality should be satisfied:

(8) $$\begin{array}{c} \frac{f_{3}}{f_{1}}\leq HC\left(1-d_{5}\right)\text{,} \end{array}$$

where HC denotes the HR cost in the previous year and *d*_5_ denotes the average rate of increase in this cost.

On the basis of the aforementioned analysis, the established multiobjective model can be expressed as follows:

(9) $$\begin{array}{c} \begin{array}{c} f_{1}=\left(E_{1}+E_{2}+E_{3}{+E}_{4}\right),\\ f_{2}=s_{1}c_{1}+s_{2}c_{2}+s_{3}c_{3}+s_{4}c_{4}-c_{5},\\ f_{3}=s_{1}c_{1}+s_{2}c_{2}+s_{3}c_{3}-{Gx}_{5}\alpha_{2}, \end{array}\\ \begin{array}{c} f_{1}=\frac{\left(E_{1}+E_{2}+E_{3}\right)}{E}\leq d_{1},\\ x_{4}\leq d_{2},\\ x_{5}\leq d_{3}, \end{array}\\ s.t\left\{\begin{array}{c} b_{11}\leq \frac{a_{1}c_{1}}{a_{1}c_{1}+a_{2}c_{2}+a_{3}c_{3}+a_{4}c_{4}}\leq b_{12},\\ b_{21}\leq \frac{a_{2}c_{2}}{a_{1}c_{1}+a_{2}c_{2}+a_{3}c_{3}+a_{4}c_{4}}\leq b_{22},\\ b_{31}\leq \frac{a_{3}c_{3}}{a_{1}c_{1}+a_{2}c_{2}+a_{3}c_{3}+a_{4}c_{4}}\leq b_{32},\\ b_{41}\leq \frac{a_{4}c_{4}}{ac_{1}+a_{2}c_{2}+a_{3}c_{3}+a_{4}c_{4}}\leq b_{42}, \end{array}\right)\\ \begin{array}{c} \frac{f_{2}}{f_{1}}\leq IF\left(1-d_{4}\right),\\ \frac{f_{3}}{f_{1}}\leq HC\left(1-d_{5}\right). \end{array} \end{array}$$

#### 3.4.3. Fuzzy Extensions

In a multiobjective model, many coefficients and parameters must be determined. Some of these parameters can be obtained from historical records such as local statistical records. For parameters with inadequate, incomplete, imprecise, or inconsistent data, domain experts can subjectively determine the values for these parameters. Because HRP involves uncertainties and great influence, each considered HR policy in this study could not be implemented realistically in the case institution. As mentioned, fuzzy programming is useful for solving programming problems involving uncertainties. Accordingly, this study incorporated fuzzy programming into the aforementioned multiobjective model to handle potential uncertainties in the selection of health-care-related HRP.

In general, the triangular fuzzy parameters, which can be expressed in terms of a triplet of crisp numbers [i.e., (*r*_1_, *r*_2_, *r*_3_), where *r*_1_ < *r*_2_ < *r*_3_], are used to describe fuzzy coefficients. The membership function of a fuzzy parameter can be expressed as follows:

(10) $$\begin{array}{c} \mu \left(x\right)=\frac{x-r_{1}}{r_{2}-r_{1}},if\;r_{1}\leq x\leq r_{2};\;\frac{x-r_{3}}{r_{2}-r_{3}},if\;r_{2}\leq x\leq r_{3};0,otherwise\text{.} \end{array}$$

Fuzzy parameters are assumed to be triangular; therefore, the fuzzy equivalent of *a* can be denoted as *ã*. Let be *x* a decision vector; *ξ* be a fuzzy vector; *f*_*i*_(*x*, *ξ*), *i* = 1, 2,…, *n*, be an objective function; and *g*_*i*_(*x*, *ξ*) be a constraint function. Therefore, the following equation can be obtained for a fuzzy multiobjective decision model:

(11) $$\begin{array}{c} \mathrm{Max}\;\left\{f_{1}\left(x,\xi \right),\ldots ,f_{i}\left(x,\xi \right),\ldots ,f_{n}\left(x,\xi \right)s.\;t.\;g_{i}\left(x,\xi \right)\leq 0,j=1,2\ldots \;p\right\}\text{.} \end{array}$$

This model can be used to solve fuzzy programming problems. Because of this model's fuzzy nature, its precision cannot be compared with that of a mathematical model. Domain experts must thus determine the expected values of the model parameters. For the triangular fuzzy parameter *ã* = (*r*_1_, *r*_2_, *r*_3_), the expected value is *ã* = 1/3 × (*r*_1_ + *r*_2_ + *r*_3_). By calculating the expected values for fuzzy parameters, experts can transform a fuzzy multiobjective model into a classic crisp MOP model, whose solution can be derived using the method described in the following section.

#### 3.4.4. Method for Solving Multiobjective Problems

In general, four types of methods are used to solve multiobjective problems: methods with no articulation of preference information, methods with a priori articulation of preference information, methods with a progressive articulation of preference information, and methods with a posteriori articulation of preference information. Solving a multiobjective problem basically involves transforming it into a single-objective problem. The most common approach for this transformation is the weighted-sum method, which involves a posteriori articulation of preferences. To illustrate the weighted-sum method, the following multiobjective problem can be used as an example:

(12) $$\begin{array}{c} \left\{f_{1}\left(x\right),\ldots .,f_{i}\left(x\right),\ldots ,f_{n}\left(x\right)\right\}s.t.\;x\in X\text{.} \end{array}$$

The first step in the weighted-sum method involves solving the following functions: max*f*_*i*_(*x*)s.t, *x* ∈ *X* and min*f*_*i*_(*x*)s.t, *x* ∈ *X*, where *i*=1, 2,…… *n*. These functions are solved to obtain the optimal value for each single-objective problem.

The second step entails applying the optimal values obtained in the first step to define new functions as follows:

(13) $$\begin{array}{c} F_{i}\left(x\right)=\frac{f_{i}^{\max}-f_{i}\left(x\right)}{f_{i}^{\max}-f_{i}^{\min}},i=1,2,\ldots .,n\text{.} \end{array}$$

The third step involves transforming the original problem into a single-objective problem as follows:

(14) $$\begin{array}{c} \min\;F\left(x\right)=w_{1}F_{1}\left(x\right)+\ldots +w_{i}F_{i}\left(x\right)+\ldots .+w_{n}F_{n}\left(x\right),s.t.\;x\in X\text{,} \end{array}$$

where *w*_*i*_ is the relative weight of the *i*th objective such that *w*_*i*_ ≥ 0, ∑_*i*=1_^*n*^*w*_*i*_=1.

The solution to the problem expressed in the preceding equation is a Pareto-optimal solution, which is satisfactory for the original problem. By using the weighted-sum method, a decision-maker can easily adjust the importance of each objective. Consider, for example, the three objectives outlined in Section 3.6.1. The parameters *w*_1_, *w*_2_, *w*_3_, *w*_4_, and *w*_5_ denote the relative weights of the objectives pertaining to health-care institution development, the patient health system, the insurance spending system, the staff assignment system, and care risk management, respectively. If the importance of the health-care institution's development must be emphasized, *w*_1_ can be set to 0.6 and *w*_2_–*w*_5_ can be set to 0.1. However, if all five objectives are considered to be of equal importance, *w*_1_–*w*_5_ are set as 1/5.

### 3.5. Model Test

According to Coyle [56], the validity of an SD model does not depend on its absolute accuracy; instead, it depends on its suitability for solving the complex and nonlinear problems. Forrester [28] also stated that an SD model developed for a complex high-order nonlinear system with numerous nodes cannot be validated using general statistical methods. These statements are valid because SD models reflect real-world situations. If some nonsignificant node relationships in an SD model are removed, the purpose of developing the model might not be achieved [49]. Considering these statements, we adopted Sterman's [49] suggestion and performed a model behavior test and model structure tests. The following model structure tests were performed using the Vensim 6.3 DSS simulation software tool: structure verification, dimensional consistency, and extreme condition tests.

In the structure verification test, we performed two interviews: one before the causal loop diagram was created and one after the flow diagram was created. By exploring the case hospital's management problems, we determined the main simulation structure required for conducting policy simulations in this study. After identifying and confirming the relationships, we performed syntax checking, single-equation checking, lookup usage checking, model checking, and multiple-equation checking by using functions of the Vensim software.

In the dimensional consistency test, we mainly evaluated whether clear and reasonable constants and node values could be calculated by unit synonyms and unit-checking tools to avoid inconsistent unit problems. The simulations conducted in this study were based on real data obtained from the case hospital; therefore, month, which is often used as the unit in models developed for selecting general human affairs strategies, was adopted as the basic unit of the developed SD model. The unit of all the nodes was set to month for consistency. Before starting the simulation procedure, we used the Vensim unit checking tool to ensure that all parameter units were consistent. The formulae and parameters are listed in Table 5. In the extreme condition test, we used two conditions to confirm whether the adopted simulation structure was correct. In the first method, the insurance income was set to 0 when the population was 0. In the second method, the care demand was set to 0 when the occupancy rate was 0.

In the model behavior test, different sets of data were used for different purposes. This test was used to determine whether the simulation results matched the real data from the case hospital. We attempted to determine whether the workload ratio and HR outflow would increase with the occupancy rate. All the simulation results were as expected and exhibited a trend of exponential growth.

## 4. Simulation and Results

Simulations for the designed system were conducted using the developed SD model. The model parameters were determined from hospital data provided by the Ministry of Health and Welfare in Taiwan, open data provided by the Taiwanese government, and information provided by the case hospital. Baseline scenarios were designed on the basis of the real revenue and nurse-patient ratios of the case hospital. We performed microcosm and macrocosm simulations in this study.

### 4.1. Policy Simulation Results Obtained with a Microcosm Model for the Case Hospital

The microcosm effects of different HR policies on the case hospital were analyzed using five practical conditions. Regarding HR outflow, primary-level health-care personnel often suggest that the standard patient-nurse ratio should be reduced. Specifically, they suggest that the number of patients requiring care should be decreased to reduce their heavy workload, which can mitigate the problem of HR outflow. Accordingly, we first simulated the effects of reducing the aforementioned ratio in the case hospital. We considered the three nursing models that are currently adopted in hospitals: primary nursing, team nursing, and functional nursing. Primary nursing is currently the most commonly used nursing model. In this model, one nurse must take care of several patients. Nurses only make plans for their patients and complete their tasks during their working hours (in this study, we assumed that three shifts exist per day and reduced the patient-nurse ratio for evaluation). Team nursing involves a group of nurses taking care of a group of patients. Different groups of patients are taken care of by nurses with different levels of experience. Job arrangements for nurses in the same group are based on their experience. We considered nurses of different levels, divided them into four groups, and performed a simulation using the same number of patients for the groups. Functional nursing is a task-centered nursing model that involves assigning specific tasks to personnel. Because some studies have indicated that the efficiency of the functional nursing model is high, we selected seven main tasks: material management, medication (injection), nursing planning, temperature, pulse, and respiration (TPR) measurement, making beds, training, and caring, as the basis for our calculations. We performed the simulation by increasing the quantity of HRs by 1.2.

The simulation results obtained for the nursing model and patient-nurse ratio are displayed in Figure 5. The care workload ratio did not decrease considerably when the patient-nurse ratio was reduced or when the functional nursing model was used. However, when the team nursing model was used, the care workload ratio was effectively reduced. These results indicate that reducing the standard patient-nurse ratio did not effectively reduce the care workload ratio. Instead, it led to uncertainty in the number of available beds, which increased administrative costs. When nurses with different experience levels work in groups, the pressure imposed on them decreases, which consequently reduces the personnel turnover rate.

In the second simulation, we increased the level of overtime, and the results are shown in Figure 6. An increase in overtime initially caused a decrease in workload. Nevertheless, the workload subsequently increased to the original level with time. Thus, the aforementioned policy was not helpful in reducing HR outflow.

In the third simulation, we adjusted the levels of experience of the nurses to increase the health-care efficiency and number of patients cared for. We simulated the effects of applying different policies, such as incentives, retention bonuses, and high salaries, for nurses with different levels of experience. We found that when the turnover rate of senior personnel was minimized, the workload did not decrease. However, when the turnover rate of personnel working in their trial period was reduced to 0, the overall HR turnover and workload decreased. This result can be used as a reference for designing salary policies in the medical field, and it contradicts the line of thinking adopted by current hospital managers. Specifically, hospital managers attempt to control HR outflow by promoting senior and advanced personnel. Moreover, they attempt to reduce the contribution of the salaries of primary-level personnel to the overall hospital cost; nevertheless, these personnel constitute a critical group of HRs providing adequate first-line health-care in a hospital. Therefore, managers should consider other policy strategies.  Figure 7 indicates that reducing the turnover rate of new employees in their trial period is the most effective policy for HR outflow reduction.

We did not consider management costs in the fourth simulation. In this simulation, we doubled the number of health-care personnel in the case hospital and then examined the corresponding effect on the workload. This examination revealed that the workload increased considerably after a short period. Therefore, the strategy of doubling the number of personnel is unsuitable for reducing HR outflow. Furthermore, as displayed in Figure 8, directly hiring an excessive number of new employees increases communication costs for senior health-care personnel, which in turn increases health-care risks.

The fifth simulation involved reducing the number of beds, and the simulation results are presented in Figure 9. A reduction in the number of beds had no effect on the nursing workload under the general health-care model. However, when we combined this policy with the policy of increasing the number of health-care personnel (i.e., when we reduced the number of beds while increasing the number of health-care personnel), the HR outflow decreased. Nevertheless, over the long term, a reduction in the number of beds resulted in increases in the occupancy rate and workload.

Various factors might influence HRP. Traditionally, predictions regarding the total HRs required in an institution are made on the basis of a single aspect. The processes adopted by managers in policy-related decision-making are simple, and their thinking can easily become linear. Examining problems involving systematic thinking is difficult. Moreover, SD modeling is highly suitable for HR policy simulations. However, as indicated in this study, the HR outflow of health-care personnel can be influenced by not only internal factors but also external factors, which include increased medical demand due to population aging in the relevant area, competition between institutions, and NHIA policies (e.g., in Taiwan, nursing fees are part of ward fees and thus receive less attention from managers). Nevertheless, SD modeling can provide some crucial insights. Accordingly, our simulation results are valuable for hospital managers. The following section describes the simulation results that were obtained by using a simple representation of the developed SD model to emphasize the relationships between the nodes of the stock flow diagram and external related systems.

### 4.2. Policy Simulation Results Obtained with a Macrocosm Model for the Case Hospital

In the area where the case hospital is located, the demand for medical services has been increasing because of the growth of the elderly population. Moreover, the development of the transportation infrastructure in the area has increased the convenience of traveling, meaning that more people can easily travel to the hospital for medical attention; this has increased personnel workload and thus aggravated the problem of insufficient medical HRs. We conducted a macrocosm simulation of Taiwan's medical resource growth by using a simplified representation of the designed SD model (Figure 10), in which we combined three objectives: hospital, insurance, and health-care HR systems to the model.

Three baseline scenarios with different rates of population growth and health-care revenues (10%, 20%, and 30% of population increase rate) were designed. The parameters of the simplified SD model were determined using statistical information obtained from Taiwan's Directorate General of Budget, accounting and statistics, and open data obtained from the Taiwan Ministry of Health and Welfare. The parameters of this model are presented in Table 6.

In multiobjective decision-making, the parameters considered (e.g., decisions related to a health-care institution's overall expenses, its insurance costs, and the workload of its care personnel) depend on the decision-maker's preferences. In this study, we assumed that the decision-maker uses fuzzy language to express uncertain quantities, and we transformed these uncertain quantities into fuzzy numbers. For example, the growth rate for each level of a health-care institution or clinic is between approximately 0.06 and 0.15 (i.e., 0.06 < *X*_*i*_ < 0.15, *i* = 1, 2, 3). Therefore, in this study, all the fuzzy coefficients were assumed to be triangular fuzzy parameters, and a multiobjective model was developed on the basis of the model described in Section 3.4. Because of constraints related to time and data collection, the scope of the macrocosm simulation was limited to western medicine; thus, data for Chinese medicine and dental medicine were excluded. Different solutions were obtained for different objective weights (Table 7). Because the first and second objectives were more important than the third objective, two weight selection methods were used. In the first method, the importance of the first and second objectives was emphasized (e.g., cases 1, 2, and 3 adjust the ratio step by step). Moreover, in the second method, the importance of the three objectives was balanced (e.g., case 3 and 4). Last, some extreme cases were also arranged (e.g., cases 5 and 6).

The macrocosm simulation results are illustrated in Figures 11–14. The proportion of health-care revenue in cases 1 and 2 changed with time (Figure 11), similar to the evaluation results obtained in the next case. Moreover, regarding the second objective, an exponential growth was observed in case 5 (Figure 12). The proportion of revenue in case 2 was slightly reduced relative to that in case 1; however, the proportion in case 2 increased considerably with time, which indicates that the insurance fee was a sensitive parameter and it alter very fast. If the current industrial structure in Taiwan remains unchanged, the insurance consumption in Taiwan would increase rapidly. In addition, the simulation results obtained when a high weight was assigned to the third objective (Figure 13) were similar to those obtained when a high weight was assigned to the first objective. However, the effect of different cases strategy was temporary, and the growth curve eventually became smooth. In case 4, the same weight was assigned to the three objectives; hence, we expected the growth rates to be consistent. However, we noted negligible differences between the simulation results obtained in Cases 4–6 (Figure 14). Accordingly, the simulation results indicate that adopting a balanced strategy for realizing multiple objectives is advantageous for health institutions.

Finally, we substituted real data into our SD overall model. When we set the same value for the GDP growth rate and population growth rate of Taiwan and considered insurance premiums to be positive, we noted that the required growth rate of the health-care in Taiwan was maintained at approximately 3.813 and that 700 care personnel were added to the workforce (approximately equal to the number of care staff members in a medium-sized medical center). This thus led to the achievement of a balance between medical demand and medical supply. These results indicate that health-care staff members in Taiwan are being overloaded at work.

Taiwan's NHI program is one of the world's best health insurance systems. A financial crisis will still happen if medical expenses get more and more increasing. Therefore, to make the best use of NHI fees, cost-saving policies regarding medical institutions' scales must be implemented. Increases in medical demand and limited income can increase the workload of medical staff members, which could predispose them to emotional risks. Accordingly, we provide the following suggestions for reducing employee workload in hospitals in the same area as the case hospital:

#### 4.2.1. Optimal Distribution of the Level of Care in the Hospital

Currently, three metropolitan hospitals and five district hospitals, all of which are acute hospitals, are located in the same area as the case hospital. This area has a large population of elderly people, is positioned by the Taiwanese government as a tourism-friendly area, and is suitable for retirement; therefore, the development of diversified long-term care systems should be promoted in this area on the basis of local residents' characteristics. The development of a subacute medical care system, such as that in the United States, or an intermediate care system, such as that in the United Kingdom, can reduce the workload of health-care personnel caused by high demands in acute hospitals.

#### 4.2.2. Development of Subsidiary Medical Institutions at Local Universities to Attract an Increasing Number of Outstanding Talents for Permanent Stay

The study interviews indicated that many doctors and other health-care personnel of the case hospital use their leave days to take degree courses or to teach in order to obtain a teaching certificate. In addition to wasting time due to commuting to their learning or teaching venues, these employees leave the case hospital after they obtain their degree. Therefore, to resolve this problem, subsidiary medical institutions can be established in local universities.

#### 4.2.3. Promotion of Health and Improvement of Self-Care Capabilities among Elderly People

The interview results indicated that in the area where the case hospital is located, changes in family structures have forced many of the elderly people to live alone, which can negatively influence their healing. The hospitals in the area should cooperate with social workers to develop diversified health promotion programs for improving residents' health awareness, health literacy, and self-care. Such programs can reduce the medical demand.

#### 4.2.4. Development of Integrated Information Platforms and Automatic Delivery Systems

Improving employees' work efficiency is the most effective strategy for reducing the pressure related to HR costs caused by increased medical demands. The central government can encourage hospitals in the considered area to increase their overall work efficiency through measures such as financial support, supporting policies, and incentive mechanisms. For example, the computerization of medical record systems can improve work efficiency. Data and interfaces from different systems should be continually integrated. Moreover, the hospitals in this area can develop a personalized health platform for residents, which can enable them to identify more people in need of medical services. They can apply the capitation payment system to reduce the overall medical demand. The automatic delivery system used in the case hospital can be adopted in other hospitals in the area to reduce employees' workload.

## 5. Conclusions and Managerial Implication

Because of advances in various forms of media, the information asymmetry between doctors and patients has decreased. However, disputes often occur between health-care personnel and patients, which can create mental pressure for health-care personnel and result in HR outflow from medical institutions. Nearly all hospitals in Taiwan are covered by the NHI program; thus, their income is limited. However, medical demands are increasing because Taiwan's elderly population is growing. In addition to medical centers and university hospitals, small and medium-sized hospitals are facing the problem of HR outflow. This phenomenon is most commonly observed among nursing staff members, for whom the workload is high but the salary is low.

Managers usually modify the HR policies of their medical institutions through trial-and-error approaches to overcome the problem caused by nursing personnel turnover. Such trial-and-error approaches can lead to the failure of HR policies, resulting in the waste of money and other resources. To overcome this problem, this study developed an SD model to simulate the effects of various HR strategies in a case hospital in different scenarios. Moreover, we constructed an SD-integrated MOP model to simulate the long-term effects of different HR strategies in the case hospital under various scenarios. This model can assist HR policymakers in medical institutions to achieve trade-offs between different objectives when attempting to reduce HR outflow.

This study has some limitations. First, data were collected from only one hospital. The scale of the developed model was reduced to cover only the field of HRs. Future studies can investigate hospitals of different levels and examine the different strategies resulting in findings between long-term care institutions and general hospitals. Moreover, the workload-related system developed for health-care staff in this study is a preliminary framework for controlling their workload. However, under the NHI system, the NHI system is more favorable to institutions that are already at a stronger position. Future studies can consider factors related to external competition from other hospitals to determine whether such factors lead to an unnatural distribution of HRs; the findings of such studies can serve as a reference for the establishment of policies in relevant institutions. Third, only fuzzy uncertainty was considered in the developed MOP model. Future studies can consider other types of uncertainty, such as stochastic uncertainty, to examine additional risk factors for HR outflow.

## Figures and Tables

**Figure 1:** Causal feedback loop diagram of the react policies about loss of care staffs. Note. P1∼P5: positive loop; N1–N9: negative loop; circle1∼circle5: strategy.

**Figure 2:** The stock-flow diagram for human resources in nursing.

**Figure 3:** The function of human resource outflow due to increase in workload.

**Figure 4:** The stock-flow diagram of the microcare staff's workload model.

**Figure 5:** Comparison evaluation results between baseline and different care models.

**Figure 6:** Comparison evaluation results between baseline and overtime policy.

**Figure 7:** Comparison evaluation results among policy for remaining differential care staffs.

**Figure 8:** Comparison evaluation results between baseline and increase manpower.

**Figure 9:** Comparison evaluation results between baseline and reduce beds.

**Figure 10:** The stock-flow diagram of the macrocare staff workload model.

**Figure 11:** Comparison results among six cases in the objective one.

**Figure 12:** Comparison results among six cases in the objective two.

**Figure 13:** Comparison results among six cases in the objective three.

**Figure 14:** Health institution growth rate after multiple objectives adjusting function.

**Table 1:** Population of the case administrative district.

Year	Birth		Death		Social increase rate		Population	Elderly rate
2000	6388	0.014	3162	0.007	−2624	−0.006	465186	0.145
2001	5487	0.012	3221	0.007	−3969	−0.009	465799	0.148
2002	5092	0.011	2935	0.006	−4319	−0.009	464107	0.152
2003	4701	0.010	3305	0.007	−2876	−0.006	463284	0.155
2004	4428	0.010	3441	0.007	−3852	−0.008	462286	0.158
2005	4098	0.009	3161	0.007	−3412	−0.007	461586	0.159
2006	3952	0.009	3221	0.007	−3025	−0.007	460426	0.16
2007	3796	0.008	2935	0.006	−1715	−0.004	460398	0.162
2008	3683	0.008	3305	0.007	−3501	−0.008	460902	0.164
2009	3683	0.008	3441	0.007	−2412	−0.005	461625	0.168
2010	3637	0.008	3544	0.008	−2266	−0.005	460486	0.173
2011	3448	0.008	3490	0.008	−1577	−0.003	459061	0.18
2012	3930	0.009	3476	0.008	−1895	−0.004	458595	0.186
2013	3531	0.008	3495	0.008	−519	−0.001	458456	0.192

Source: budget, accounting and statistics department of local county; P.S.: birth rate: means the total number of births per 1000 of population each year; young age means population by age of 0–14; working age means population by age of 15–64; elderly means population by age of 65 and over; social increase rate means the immigrant rate subtracting the emigrant rate; total population = (young age + working age + elderly) *∗* (1 + social increase rate).

**Table 2:** Medical visits and points of case hospital for revenue subsector.

Year/month		Hospital outpatient		Hospital inpatient	
		Visits	Medical points	Visits	Medical points
101	1	56722	164,447,252	4,436	165,710,659
101	2	44812	108,866,638	3,882	118,505,577
101	3	47992	128,145,124	4,271	143,449,344
101	4	55516	161,820,331	4,313	173,307,089
101	5	54391	159,923,394	4,363	163,446,223
101	6	46246	125,912,544	4,174	148,963,647
101	7	58280	173,265,634	4,458	173,488,691
101	8	53153	152,568,364	4,372	155,011,434
101	9	46291	128,705,569	4,117	142,019,141
101	10	58660	177,711,212	4,304	166,300,818
101	11	51426	144,346,940	4,192	157,847,699
101	12	54385	159,835,276	4,313	170,175,597
102	1	52916	147,071,264	4,995	209,700,289
102	2	53858	135,073,360	4,276	156,556,231
102	3	55692	152,597,484	4,762	204,766,443
102	4	61262	169,234,139	4,792	206,670,431
102	5	62737	166,681,236	5,238	213,385,929
102	6	57035	147,975,918	4,301	165,745,638
102	7	63862	173,854,512	4,640	176,675,969
102	8	59569	153,677,310	4,261	162,280,972
102	9	60040	157,683,212	4,201	162,262,866

**Table 3:** A comparison of each year of nursing staff outflow.

Year	Number of staffs	Average staff turnover rate
2009	324	0.027
2010	325	0.045
2011	323	0.047
2012	322	0.05
2013	325	0.052
2014	314	0.081

**Table 4:** List of parameters.

Notation	Explanation
*f*_1_	Objective related to a health-care institution's revenue
*f*_3_	Objective related to human resource planning
*G*_2_	Patient care revenues
*E*1	Revenue of hospital
*E*3	Revenue of district hospital
*x*_1_	Growth rate of hospital
*x*_3_	Growth rate of hospital
*x*_5_	Proportion of investment in the remaining staff
*C*_1_	Global budget for western medicine consumption
*C*_3_	Global budget for dental medicine consumption
*C*_5_	Reduction in hospital expenses after the implementation of the global budget
*s*_*i*_	Consumption coefficient of fee *i* to human resource loss
*α*_1_	Restrictive impact factor coefficient for the global budget system
*f*_2_	Objective related to the insurance system
*G*_1_	Patient care revenue under health insurance
*G*_3_	Nonpatient revenue
*E*2	Revenue of a metropolitan hospital
*E*4	Revenue of a clinic
*x*_2_	Growth rate of a metropolitan hospital
*x*_4_	Administration fee in the global budget
*C*_2_	Global budget of western primary medicine consumption
*C*_4_	Global budget of Chinese medicine consumption
*a*_*i*_	The exhausted of care staff equivalent transformation coefficient of the insurance of fee *i*
*e*_*ij*_	Consumption coefficient of fee *i* per unit of output for the *j*th hospital level
*α*_2_	Implement impact factor on coefficient of human loss policy

**Table 5:** The formula using the software ‘Vensim' to simulate the talent retention policy model.

Level/rate	Formula or default observations
Income of institution	INTEG (insurance income + noninsurrance income + nonmedical insurance) − cost − global budget cost
Scheduling parameter	0.2
Total number of staffs	Number of trial staffs + number of junior staffs + number of advanced staffs + number of staffs planning to resign + number of expert staffs
Number of trial staffs	INTEG (hire − qualification − number of trial staffs resigned)
Number of junior staffs	INTEG (Qualification − proficiency)
Number of advanced staffs	INTEG (Proficiency − contract − number of junior staffs resigned)
Number of staffs planning to resign	INTEG (number of junior staffs resigned + number of advance staffs resigned + number of senior staffs resigned- number of staffs confirmed to resign)
Number of expert staffs	INTEG (contract- position adjustment − number of expert staffs resigned)
Qualification	(Number of trial staffs − number of trial staffs resigned)
Time required for qualification	3
Proficiency	Number of junior staffs/time required for proficiency
Time required for proficiency	6
Contract	(Number of advance staffs − number of junior staffs resigned)/contract period
Contract period	24 (2 year)
Position adjustment	Number of senior staffs/time required for position adjustment
Time required for position adjustment	24
Number of trial staffs resigned	Number of trial staffs *∗* trial staff turnover rate
Number of junior staffs resigned	Number of junior staffs *∗* junior staff turnover rate
Number of staffs confirmed to resign	Number of staffs planning to resign/time required for staffs confirmed to resign
Number of senior staffs resigned	Number of senior staffs *∗* senior staff turnover rate
Trial staff turnover rate	0.3
Junior staff turnover rate	0.5
Senior staff turnover rate	0.3
Confirmed time to leave office	1
Total number of care staffs	Number of trial staffs + numbert of junior staffs + numbert of senior staffs + number of staffs planning to resign + numbert of expert staffs
Time required for reassignment	1
Time required for hiring	3
Weighted total number of people	MAX (number of trial staffs *∗* weight for trial staffs + number of junior staffs *∗* weight for junior staffs + number of advance staffs *∗* weight for senior staffs + number of prepared to leave job *∗* weight for staffs prepared to leave job + number of expert staffs *∗* weight for advanced and senior staffs, 0)
Weight for trial staffs	−0.1
Weight for staffs prepared to leave job	0.9
Weight for advanced and senior staffs	1.2
Weight for junior staffs	0.8
Influence of staffs leaving office	1⟶4⟶7⟶8 > 9 (trial staffs⟶senior staffs⟶advanced staffs⟶senior staffs⟶expert staffs)
Care hours required	Person-times of hospitalization *∗* seriousness of disease
Person-times of hospitalization	Number of hospitalized patients *∗* 24/3 *∗* (1/Day shift nurse-patient parameter + 1/Evening shift nurse-patient parameter + 1/Overnight shift nurse-patient parameter) *∗* parameter for transfer or discharge
Parameter for transfer or discharge	0.9
Seriousness of disease	1.5
Supplied hours	Weighted total number of people *∗* 8 *∗* shifts *∗* average overtime parameter
Shifts	22
Workload ratio	XIDZ (care hours required, supplied hours, 50)
Average workload ratio	INTEG (different in workload ratio, 1)
Different in workload ratio	Workload ratio *∗* average workload ratio
Change in workload ratio	Different in workload ratio/responding time
Responding time	1
Day shift nurse-patient parameter	8 *∗* workload parameter
Evening shift nurse-patient parameter	10 *∗* workload parameter
Overnight shift nurse-patient parameter	12 *∗* workload parameter
Workload parameter	MIN (average workload ratio, 1.5)
Overtime parameter	MIN (average workload ratio, 2)
Average overtime parameter	INTEG (change rate of overtime, 1)
Difference in overtime parameter	Overtime parameter-average overtime parameter
Change rate of overtime	Difference in overtime parameter/time required to change shift
Time required to change shift	6
Influential coefficient of overtime	Influential function of overtime (ovetime parameter)
Resignation of trial staffs	Number of trial staffs *∗* MIN (trial staff turnover rate *∗* influential function for trial staffs, 1)
Resignation of junior staffs	Number of advanced staffs *∗* MIN (junior staffs turnover rate *∗* influential function for junior staffs, 1)
Resignation of senior staffs	Number of senior staffs *∗* MIN (senior staffs turnover rate *∗* influential function for senior staffs *∗* influential function for senior staffs, 1)
Number of beds available	INTEG (number of open beds − number of beds reduced)
Number of open beds	IF THEN ELSE (difference in number of beds ≥ 0, difference in number of beds/time required to open beds, 0)
Number of beds reduced	IF THEN ELSE (difference in number of beds < 0, MIN (−difference in number of beds/time required to reduce beds, number of beds available, 0)
Time required to open beds	3
Time required to reduce beds	9
Difference in number of beds	Approved number of beds-number of beds available
Estimated number of beds	SMOOTH (number of beds affordable, 3)
Number of beds affordable	MIN (total number of care staffs *∗* patient-nurser standard, approved number of beds)
Approved number of beds	750
Patient-nurser standard	2.5
Target number of nursing staffs	Number of beds affordable/Patient-nurser standard
Number of hospitalized patients	Delay (number of beds available *∗* 30 *∗* occupancy rate, 1)
Occupancy rate	70 (including reduce beds)
Effect of implementation of technology	Time required for proficiency *∗* weight for each staffs
Coefficient for administrative tasks	MIN (average workload ratio, 1.2)

**Table 6:** Data of the coefficients.

Notation	Value	Unit
*G*_1_	64028.72	10^5^ NT$/month
*G*_3_	6259.06	10^5^ NT$/month
*a*_2_	13	%
*s*_1_	42.75	%
*s*_3_	0.05	%
*e*_21_	16.46	%
*e*_12_	88.47	%
*e*_32_	0.42	%
*e*_23_	8.4	%
*G*_2_	9087.46	10^5^ NT$/month
*a*_1_	76	%
*a*_3_	10	%
*s*_2_	52.25	%
*e*_11_	83.14	%
*e*_31_	0.4	%
*e*_22_	11.11	%
*e*_13_	91.6	%
*e*_33_	0.1	%

**Table 7:** Trade-offs between the objectives.

Case number	*fw*_1_	*fw*_2_	*fw*_3_
Case 1	0.9	0.05	0.05
Case 2	0.8	0.1	0.1
Case 3	0.5	0.3	0.2
Case 4	0.33	0.33	0.33
Case 5	0.1	0.8	0.1
Case 6	0.1	0.1	0.8

## Data Availability

The data used to support the finding of this study are included within the article.
